# Senescence Osteoblast-Derived Exosome-Mediated miR-139-5p Regulates Endothelial Cell Functions

**DOI:** 10.1155/2021/5576023

**Published:** 2021-04-15

**Authors:** Qing Lu, Hao Qin, Haitao Tan, Cansen Wei, Xinni Yang, Jinqiao He, Weibing Liang, Jing Li

**Affiliations:** ^1^Department of Physiology, Guangxi Medical University, Nanning, China; ^2^Guangzhou Kangda Vocational Technical College, Guangzhou, China; ^3^Department of Orthopedics, Eighth Affiliated Hospital, Guangxi Medical University, Guigang, China; ^4^Key Laboratory of Longevity and Aging-Related Diseases, Ministry of Education, Nanning, Guangxi, China

## Abstract

The pathogenesis of osteoporosis is considered extremely intricate. Osteoblast differentiation and angiogenesis can greatly affect bone development and formation, given their coupling role in these processes. Exosome-mediated miRNA regulates cellular senescence, proliferation, and differentiation. However, whether senescent osteoblasts can regulate the senescence of vascular endothelial cell by miRNA through exosomal pathway remains unclear. In this study, senescent osteoblasts could regulate endothelial cell function, promote cell senescence and apoptosis, and decrease cell proliferation via exosomal pathway. miR-139-5p showed high expression in senescent osteoblasts and their exosomes. After senescent osteoblast-derived exosome treatment, miR-139-5p was also upregulated in endothelial cells. Furthermore, transfection of miR-139-5p mimic promoted the senescence and apoptosis of vascular endothelial cells and inhibited their proliferation and migration, whereas transfection of miR-139-5p inhibitor rescued the effect of D-galactose. Using double luciferase assay, TBX1 was confirmed to be a direct target gene of miR-139-5p. In conclusion, senescent osteoblast-derived exosome-mediated miR-139-5p regulated endothelial cell function via exosomal pathway. Our study revealed the role of osteoblast-derived exosomes in the bone environment during aging, providing a clue for inventing a new target therapy.

## 1. Introduction

Considering the close relationship between osteogenesis and angiogenesis, an increasing number of studies started investigating the relationship between osteoporosis, which is a very common disease, and angiogenesis [1]. The widely accepted relationship between these two is that the reduction of angiogenesis causes osteoporosis and the promotion of local angiogenesis alleviates it [2] and the bone matrix can secrete proangiogenic endothelial cell factor and promotes angiogenesis in reverse, which provides the necessary nutrients and regulators for osteogenesis [3–5]. The degree of osteoporosis indeed accelerates decreased angiogenesis, but it does not provide a more in-depth understanding between the mechanisms of osteoporosis and angiogenesis.

Exosomes are 30-150 nm sized vesicles that are widely distributed in various body fluids. The exosome membrane primarily comprises lipids and proteins that carry a variety of proteins, nucleic acids, microRNA (miRNA), and mRNA, which can be absorbed by other cells in order to regulate recipient cells [6]. miRNAs are defined as noncoding, single-stranded RNA molecules of about 22 nucleotides in length that mediate posttranscriptional gene silencing by binding to the 3′-UTR or open reading frame region of target mRNA, which can affect the generation of many protein-coding genes identified to be participating in the regulation of several organismal life activities, such as cell proliferation, differentiation, migration, and even disease progression [7]. Owing to the transport capabilities of vesicles, the role of miRNAs in exosomes is being increasingly appreciated.

It has been previously demonstrated that osteoblast-secreted vascular endothelial growth factor (VEGF) promoted angiogenesis, whereas vascular endothelial cells improved osteoblast function [8]. We speculate that endothelial cell could affect osteoblasts and then accelerate osteoporosis if osteoblasts can regulate angiogenesis during the aging process. However, how osteoblasts affect angiogenesis during aging process is still unclear. In this study, with an ultimate goal of providing novel insights on osteoporosis therapy, we observed the changes of vascular endothelial cell after cocultured with senescent osteoblasts and miR-139-5p mimic or inhibitor, in order to explore how osteoblast exosome-derived miRNA affects vascular endothelial cell during aging process, providing new ideas for osteoporosis therapy.

## 2. Materials and Methods

### 2.1. Cell Culture and Transfection

BALB/c mice of 5–7 days age (Animal Center, Guangxi Medical University, China) were used to extract primary osteoblasts via enzyme digestion (Type II Collagenase, Gibco, CA, USA). Primary osteoblasts were identified using alkaline phosphatase staining (Beyotime, Shanghai, China). Vascular endothelial cells were obtained from Aolu Company (Shanghai, China). These were cultured in MEM*α* medium (Gibco, CA, USA) supplemented with 10% fetal bovine serum (Gibco, CA, USA) and 100 U/ml each of penicillin and streptomycin (Gibco, CA, USA). Cells were maintained in a thermostatic incubator with 5% CO_2_ at 37°C. In the coculture system, osteoblasts were seeded in the upper chamber of a Transwell chamber (Corning, USA) at a density of 2.0 × 105 cells/ml and endothelial cells were inoculated in 6-well plates (Corning, USA) at a density of 1.0 × 105 cells/ml. The Transwell chambers were placed into plates after both cell types reached adherent growth densities of 50%. miR-139-5p mimic and inhibitor with their negative controls were synthesized using riboFECT CP (RiboBio, Guangzhou, China) and transfected into endothelial cells using riboFECT CP reagents, following the manufacturer's instructions.

### 2.2. Senescence *β*-Galactosidase (SA-*β*-Gal) Assay

SA-*β*-gal assay was performed using a *β*-galactosidase staining kit (Beyotime, Shanghai, China), cultured cells were fixed at room temperature for 5 min in 2% formaldehyde and 0.2% glutaraldehyde, and then stained with SA-*β*-gal staining solution at 37°C overnight, and images were captured using a microscope digital camera (Olympus). The percentage SA-*β*-gal-positive cells were calculated with ImageJ.

### 2.3. Cell Apoptosis Assay

Once cell density reached about 50%, 0.5% Hoechst 33258 staining solution (Beyotime, Shanghai, China) and dye were added for 5 minutes and then discarded. After placing a drop of antifluorescence sealing liquid on the cells, the blue-stained nucleus could be detected using a fluorescence microscope, with an excitation wavelength of about 460 nm. The TUNEL (TdT-mediated dUTP nick-end labeling) cell apoptosis detection reagent (Zhongshan Jinqiao, Beijing, China) was prepared according to the instruction manual and then added to the climbing tablet to perform both 3,3′-diaminobenzidine (DAB) and hematoxylin staining.

### 2.4. Cell Proliferation Assay

The SP staining kit (Zhongshan Jinqiao, Beijing, China) and Ki-67 cell proliferation detection kit (Sangon Biotech, Shanghai, China) assay were used to detect cell proliferation. Cells cultured to a density of approximately 70% were used. The cells were immobilized on glass slides before they were incubated with the antibodies and added onto the climbing tablet to perform DAB and hematoxylin staining.

### 2.5. RNA Isolation and Quantitative Reverse Transcription Polymerase Chain Reaction (RT-PCR)

Total RNA from the cells was isolated using TRIzol reagent (Invitrogen, CA, USA) according to the manufacturer's instructions. Reverse transcription converted the RNA into cDNA, according to the microRNA First-Strand cDNA Synthesis Kit (Sangon Biotech, Shanghai, China) instructions. RT-PCR reactions were performed using SYBR Green PCR Master Mix (Applied Biosystems). The miRNA expression levels and target gene mRNA were standardized to U6 and glyceraldehyde 3-phosphate dehydrogenase, respectively. The results were analyzed using the 2^−ΔΔCt^ method. The primer sequences used in this study are described in Table 1.

### 2.6. Exosome Isolation, Separation, and Reverse Transcription

Exosomes in osteoblast cell culture supernatant were isolated using an SBI ExoQuick-TC ULTRA EV Isolation Kit (System Biosciences, USA). Separation and reverse transcription of exosomes into cDNA were performed by using an SBI Seramir Exosome RNA Amplification Kit (System Biosciences, USA) and Cel-miR-39-3p standard RNA (RiboBio, Guangzhou, China) as external references. RT-PCR was performed to detect RNA expression in exosome using a FastStart Universal SYBR Green Master (ROX) kit (Roche, Germany).

### 2.7. Transmission Electron Microscopy (TEM)

Onto sealing films, 5 *μ*l of purified exosomes was dropped; the carbon-coated copper mesh was placed on the droplets floating. Next, 20 *μ*l of 1% phosphotungstic acid-staining droplet was stained on the sealing film for 30 s, and then, the excess liquid was drained; the sealing film was then dried, and exosomes were observed by standard TEM with a Philips CM120 microscope.

### 2.8. Nanoparticle Analysis

The extracted exosomes were diluted to 800-1000 ml with phosphate-buffered saline and mixed evenly with a vortex mixer and measured with Nanosight NS300 (Malvern, Britain). Sample was injected thrice for 30 s each time. NTA2.3 analysis software was used for data analysis.

### 2.9. Cell Migration Experiment

A well plate with an 8 *μ*m pore size Transwell chamber (Corning, USA) was used in measuring cell migration. The cell density was adjusted to 2 × 10^5^ cells/ml; then, 500 *μ*l of cell suspension was incubated into the upper chamber, and 750 *μ*l of the medium with serum was added into the lower chamber. After 12 h culture, the cells were fixed with POM for 15 min and then stained with 500 *μ*l of 0.1% crystal violet for 30 min. Photo counting was then performed using an inverted microscope.

### 2.10. Wound Healing Assay

Cells in 6-well plates with a density of about 5 × 10^5^ cells/well were treated with 20 *μ*g/ml mitomycin (TCI, Shanghai, China) for 3 hours. Artificial wounds were created by scratching using 10 *μ*l pipette tips and then incubated with serum-free medium. Photos were taken of the same location at 0 and 24 hours. ImageJ software was used to analyze the scratch area.

### 2.11. Western Blot

Cells were lysed using a RIPA buffer (Thermo Fisher Scientific, USA) to a protein separation of 10% SDS polyacrylamide gel. The proteins were then transferred onto PVDF membranes. First antibodies diluted with blocking solution were added and incubated overnight at 4°C, followed by incubation with either HRP-labeled sheep anti-rabbit secondary antibodies or HRP-labeled sheep anti-mouse secondary antibodies. The PVDF film was sensitized, developed, and fixed using an X-ray film in an anechoic chamber. Primary antibodies, CD9, CD63, TSG101, and calnexin (all from Abcam), were then used.

### 2.12. Dual-Luciferase Assay

The TBX1 3′-UTR wild-type (WT) and mutated (MUT) sequences of the target gene, TBX1, were cloned into the pSICheck-2 plasmid. Next, 293 T cells were incubated into 96-well plates. Objective plasmids and mutant plasmids were mixed with miRNA mimic and scrambled RNA as a negative control, respectively. Lipofectamine 2000 transfection reagent was added. Cells were collected after 48 h of transfection. The manufacturer's instructions were followed for the Dual-Luciferase System Kit (Promega, USA).

### 2.13. Statistical Analysis

All of our statistical tests for this research were performed using SPSS 25.0 software (Chicago, IL, USA). Graphs were constructed using GraphPad Prism 5 software (La Jolla, CA, USA). The *t*-test and one-way analysis of variance were used to estimate the differences between groups when appropriate. When a statistical difference was determined, the asterisk symbol was used to represent *p* < 0.05, whereas two asterisks were used to represent *p* < 0.01.

## 3. Results

### 3.1. D-Galactose Induced Senescence of Osteoblasts

Cells that emerged from the bone fragments on different days could be clearly observed under a microscope, as the cells adhered to the wall and were determined to gradually increase after 3 days, having a fusiform or irregular polygon shape (Figure 1(a)). Osteoblasts cultured in vitro were able to synthesize large amounts of alkaline phosphatase. The successful extraction of osteoblasts was confirmed by performing the alkaline phosphatase staining (Figure 1(b)). To the establishment of senescence cellular model, the osteoblasts were induced by D-galactose (D-gal). After *β*-galactosidase senescence staining and aging-related gene expression analysis, D-galactose treatment increased the number of senescence positive cells and the mRNA expression of p21 and p53 (Figures 1(c) and 1(d)), which further indicated that treatment with D-galactose induced senescence of endothelial cells.

### 3.2. Changes of Endothelial Cell Function in Coculture System

To assess whether coculture endothelial cells with senescent osteoblasts can influence endothelial cell function, Transwell model was used to explore the role of osteoblast-derived exosome in endothelial cell phenotype. The results showed that the senescence and apoptosis positive rate increased and the cell proliferation rate decreased in the endothelial cells cocultured with senescent osteoblasts (Figures 2(a), 2(b), and 2(c)). However, the senescence positive rate and apoptosis slowed down and the proliferation rate enhanced in the endothelial cells cocultured with the senescent osteoblast+GW4869 group indicated that senescence osteoblasts effect on endothelial cell function through exosome pathway (Figures 2(a), 2(b), and 2(c)).

### 3.3. miR-139-5p Was Upregulated in Osteoblast-Derived Exosome

Aging-related miRNAs were screened via bioinformatics analysis and previous studies. The qRT-PCR results showed that miR-139-5p expression increased in senescent osteoblasts, but not in senescent vascular endothelial cells (Figure 3(a)). However, the relative expression increased in vascular endothelial cells after coculture with senescent osteoblasts (Figure 3(b)). Exosomes in osteoblast cell culture supernatant were isolated and showed similar morphology, size, and number as a previous report [9] (Figures 3(c) and 3(d)). Western blot assay further verified that the exosome marker proteins, TSG-101, CD63, and CD81, were enriched in exosomes (Figure 3(e)). Furthermore, the increased miR-139-5p level was confirmed in senescent osteoblast exosomes (Figure 3(f)). Simultaneously, the senescent osteoblast-derived exosomes could accelerate the senescence and apoptosis of endothelial cells (Figures 3(g) and 3(h)).

### 3.4. miR-139-5p Accelerated Senescence and Apoptosis of Endothelial Cell

To explore the mechanism of miR-139-5p expression regulating the endothelial cell functions, miR-139-5p expression was overexpressed or inhibited by miR-139-5p mimic or inhibitor transfection and transfection efficacy was tested (Figure 4(a)). The potential influence of miR-139-5p on endothelial cell functions was investigated by *β*-galactosidase senescence staining and apoptosis assay, which showed that the senescence (Figure 4(b)) and apoptosis positive rate of endothelial cells increased after miR-139-5p mimic transfection. However, the inhibition of miR-139-5p expression could recover senescence and apoptosis ability (Figure 4(c)) of vascular endothelial cells. Collectively, miR-139-5p could promote the apoptosis and senescence of vascular endothelial cells.

### 3.5. miR-139-5p Suppressed the Proliferation and Invasion of Endothelial Cells

Cell wound healing assay found that the number in the miR-139-5p mimic group was higher than that in the NC-mimic group (Figure 5(a)), while miR-139-5p inhibitor could increase number in senescent endothelial cells. Transwell assay showed the number of endothelial cells having migrated through the Matrigel gel, and the lower layer of the filter decreased after treatment with miR-139-5p mimic and increased when senescent endothelial cells were treated with miR-139-5p inhibitor (Figures 5(b) and 5(d)). Ki67 proliferation staining assay showed that miR-139-5p mimic inhibited endothelial cell proliferation (Figure 5(c)). In contrast, the inhibition of miR-139-5p expression enhanced the proliferation (Figure 5(e)) ability of endothelial cells compared with the D-gal-induced senescence group. These suggested that miR-139-5p suppressed the proliferation and invasion of endothelial cells; however, inhibition of miR-139-5p could accelerate cell proliferation and invasion.

### 3.6. TBX1 Is a Potential Target of miR-139-5p

Through bioinformatics analysis, we screened out TBX1 as the potential target gene of miR-139-5p using high binding sites at the intersection of TargetScan, miRBase, and miRDB bioinformatics databases (Figures 6(a) and 6(b)). Furthermore, TBX1 expression was verified using qRT-PCR. The expression of TBX1 mRNA was significantly decreased in the endothelial cells with miR-139-5p overexpression, but increased in the endothelial cells with low miR-139-5p expression (Figure 6(c)). Relationship between miR-139-5p and TBX1 mRNA in endothelial cells was analyzed, and it was found that there was a negative correlation between miR-139-5p and TBX1 mRNA (Figure 6(d)). Double luciferase report showed that the fluorescence value of the miR-139-5p WT cotransfection group was significantly lower, whereas the fluorescence value of the miR-139-5p/WT cotransfection group was no different than that of the NC group (Figure 6(e)), which suggested that TBX1 was a direct target gene of miR-139-5p.

## 4. Discussion

In the present study, we demonstrated that the senescent osteoblast-derived exosome-mediated miR-139-5p regulates vascular endothelial cells functions. These findings highlight a novel mechanism of osteoblasts accelerating the change of endothelial cell during aging. Upon release from osteoblasts cells, exosomes distribute in tissue space and exert biological function remotely. This feature makes it possible for osteoblasts to influence endothelial cells without direct contact during osteoporosis.

Exosomes are considered to be present in almost all biological fluids, enriched with numerous microstructures comprising of cholesterol and sphingomyelin [10–12]. Exosomes contain various nucleic acids, including mRNA, miRNA, and other noncoding RNA [13]. Several studies have also confirmed that miRNAs can be present stably in numerous body fluids. The miRNA in these body fluids can enter the exosome vesicles or bind to AGO2 proteins on the external surface of the vesicles [6, 14–18]. However, exosomes are considered to be more efficient at transportation than other binding models, earning exosome miRNA increasing attention lately. Exosome information transmission through microcirculation is considered to be the third mode of cell-to-cell communication, which is an important as the process of cell contact signal transmission and soluble molecular signal transmission [19–22]. In the present study, we demonstrated that the endothelial cells cocultured with senescent osteoblasts showed increased senescence and apoptosis ability and decreased proliferation activity through the exosomal pathway.

Previous studies have shown that the exosome-mediated miRNAs play critical roles in various physiological and pathological processes of endothelial cell. One such recognized is the dendritic cell-mediated miR-146a contributed to protect HUVECs through inhibiting interleukin-1 receptor-associated kinase [23]. A previous study has reported that smooth muscle cell-derived exosome-mediated miR-155 induced endothelial injury and promoted atherosclerosis [24]. In this study, miR-139-3p was upregulated in senescent osteoblast and senescent osteoblast-derived exosome and these exosomes could promote the senescence and apoptosis ability of endothelial cells indicating that senescent osteoblast-derived exosome-mediated miR-139-5p affects vascular endothelial cell functions.

miRNA binds to multiple mRNA sites and plays a regulatory role in different physiological or pathological processes. Agosta et al. found that miR-139-5p promotes aggressiveness by targeting N-myc downstream-regulated gene family members in adrenocortical cancer. Moreover, miR-139-5p can suppress cell proliferation and chemotherapy resistance of non-small-cell lung cancer by inhibiting RRM2. miR-139-5p can inhibit aerobic glycolysis, cell proliferation, migration, and invasion in hepatocellular carcinoma via regulating ETS1. miR-139-5p can also inhibit the growth of hepatocellular carcinoma by targeting SPOCK1 [25–28]. In our study, we found that TBX1 is a potential target mRNA of miR-139-5p. TBX1 is mainly involved in the process of vascular differentiation and maturation, serving a crucial role in cardiovascular morphogenesis [29]. Studies in mice have confirmed that TBX1 can activate VEGFR3 in endothelial cells and affect the angiogenesis process by negatively regulating angiogenesis through the DLL4/Notch1-VEGFR3 regulatory axis [30]. Other studies have shown that the conditional deficiency of TBX1 in endothelial cells causes widespread lymphangiogenesis defects in mouse embryos and perinatal death [31]. These studies suggest that TBX1 may be involved in the regulation of aging and apoptosis of some cells or tissues. These indicated that senescent osteoblast exosome-delivered miR-139-5p is a potential regulatory pathway for endothelial cell senescence by targeting TBX1, which might be an important mechanism for osteoblast regulating endothelial cell function during osteoporosis. This study elucidates a novel cellular and molecular pathway that influences miR-139-5p expression in osteoblasts, which could lead to the development of new therapeutic approaches and provide novel insights into angiogenesis pathophysiology in osteoporosis.

## 5. Conclusion

We discovered that senescent osteoblast-derived exosome-mediated miR-139-5p regulates vascular endothelial cell functions. Mechanistically, miR-139-5p was upregulated in osteoblast during aging. Senescent osteoblast-derived exosome-mediated miR-139-5p and exosomal miR-139-5p could promote senescence and apoptosis, and inhibit proliferation and invasion of endothelial cells via target TBX1. As the change of angiogenesis affects the osteoporosis process, this study provided novel insights and therapeutic targets for the prevention and treatment of osteoporosis.

## Figures and Tables

**Figure 1:** Establishment of primary osteoblast senescence model. (a) The condition of cells emerging from bone fragments under different days. (b) Observation of alkaline phosphatase staining in primary cells. (c) Analysis of *β*-galactosidase senescence staining in osteoblasts treated with D-gal for 48 h and quantitative analysis (^∗∗^*p* < 0.01). (d) Expression of p53 and p21 genes in osteoblasts. After D-gal induction (^∗∗^*p* < 0.01).

**Figure 2:** Biological function of endothelial cells in coculture model. (a) *β*-Galactosidase senescence staining of endothelial cells cocultured with osteoblasts and quantitative analysis (∗∗ means comparison with the control group, *p* < 0.01; ## means comparison with the model, *p* < 0.01). (b) Apoptosis staining of Hoechst endothelial cells after coculture with osteoblasts and quantitative analysis (∗∗ means comparison with the control group, *p* < 0.01; ## means comparison with the model, *p* < 0.01). (c) Proliferation and staining of ki67 endothelial cells after coculture with osteoblasts and quantitative analysis (∗∗ means comparison with the control group, *p* < 0.01; ## means comparison with the model, *p* < 0.01).

**Figure 3:** Effect of osteoblast exosome-derived miR-139-5p on the biological function of vascular endothelial cells. (a) Expression of related miRNA in two types of cells treated by D-gal for 48 h. (b) Expression of miR-139-5p in vascular endothelial cells in the coculture system (∗∗ means comparison with the control group, *p* < 0.01; # means comparison with the model, *p* < 0.05). (c) Electron microscope scanning of exosome-isolated osteoblast cells and (d) particle size analysis of exosome western blot analysis (e) of exosome-enriched proteins (CD9 (22-25 kDa) and CD63 (26 kDa)) and the key proteins for miRNA function (TSG101 (45 kDa) and calnexin (90 kDa)). (f) Levels of miR-139-5p in exosomes isolated from the control and senescence groups of osteoblast cells were determined by qRT-PCR analysis (^∗∗^*p* < 0.01). (g) Senescence staining of vascular endothelial cells by the control and senescence groups of osteoblastic exosomes and quantitative analysis (^∗∗^*p* < 0.01). (h) Staining of the control and senescence groups of osteoblastic exosomes on apoptosis of vascular endothelial cells and quantitative analysis (^∗∗^*p* < 0.01).

**Figure 4:** Effects of miR-139-5p on the senescence and apoptosis of vascular endothelial cells. (a) Expression of miR-139-5p after transfection with miR-139-5p mimic and inhibitor in endothelial cells (^∗∗^*p* < 0.01). (b) Senescent staining, Hoechst apoptosis staining, and TUNEL apoptosis staining of vascular endothelial cells after miR-139-5p mimic treatment and quantitative analysis (^∗∗^*p* < 0.01). (c) Senescent staining, Hoechst apoptosis staining, and TUNEL apoptosis staining of senescent vascular endothelial cells induced by D-gal after miR-139-5p inhibitor treatment and quantitative analysis (^∗∗^*p* < 0.01).

**Figure 5:** Effects of miR-139-5p intervention on the migration and proliferation of vascular endothelial cells. (a) Wound healing assay regarding endothelial cell death with miR-139-5p intervention and quantitative analysis (^∗∗^*p* < 0.01). (b) Transwell migration and (c) ki67 proliferation staining of vascular endothelial cells after miR-139-5p mimic intervention and quantitative analysis (^∗^*p* < 0.05). (d) Transwell migration and (e) ki67 proliferation staining of senescent vascular endothelial cells induced by D-gal after miR-139-5p inhibitor intervention and quantitative analysis (^∗^*p* < 0.05).

**Figure 6:** TBX1 could be one of the potential targets of miR-139-5p. (a) Three differently expressed target genes of miR-139-5p were integrated from TargetScan and miRDB databases. (b) TBX1 was one of the intersections of miR-139-5p-associated gene targets. (c) Expression of TBX1 mRNA in endothelial cells transfected with miR-139-5p (^∗^*p* < 0.05, ^∗∗^*p* < 0.01). (d) Pearson analysis of the relationship betweenTBX1 and miR-139-5p expression. (e) The predicted binding site of miR-326-3p target gene TBX1 and dual-luciferase assay verified the targeted relationship between TBX1 and miR-139-5p.

**Table 1:** Primer sequence.

Primer name	Primer sequence
p53	F: 5′-AGTCCTTTGCCCTGAACTGC-3′ R: 5′-GCGGATCTTGAGGGTGAAAT-3′
p21	F: 5′-TGGACCTGTCACTGTCTTGT-3′ R: 5′-TCCTGTGGGCGGATTA-3′
GAPDH	F: 5′-GGTTGTCTCCTGCGACTTCA-3′ R: 5′-TGGTCCAGGGTTTCTTACTCC-3′
TBX1	F: 5′-CACCAAGGCAGGCAGACGAATG-3′ R: 5′-CTACGGGCACAAAGTCCATGAGC-3′
mmu-miR-139-5p	F: 5′-TCTACAGTGCACGTGTCTCCAG-3′

## Data Availability

The data used to support the findings of this study are included within the article.
